The article "High Detection Rate of HIV Drug Resistance Mutations among Patients Who Fail Combined Antiretroviral Therapy in Manaus, Brazil" was published in 2021. Journal: Biomed Res Int.

# High Detection Rate of HIV Drug Resistance Mutations among Patients Who Fail Combined Antiretroviral Therapy in Manaus, Brazil

**DOI:** 10.1155/2021/5567332

**Published:** 2021-06-08

**Authors:** Yury Oliveira Chaves, Flávio Ribeiro Pereira, Rebeca de Souza Pinheiro, Diego Rafael Lima Batista, Antônio Alcirley da Silva Balieiro, Marcus Vinicius Guimarães de Lacerda, Paulo Afonso Nogueira, Monick Lindenmeyer Guimarães

**Affiliations:** ^1^Laboratório de Diagnóstico e Controle de Doenças Infecciosas na Amazônia (DCDIA), Instituto Leônidas e Maria Deane (ILMD)–Fiocruz Amazônia, Manaus CEP 69.057-070, Brazil; ^2^Fundação de Medicina Tropical Dr. Heitor Vieira Dourado, Instituto de Pesquisa Clínica Carlos Borborema, Manaus, Amazonas CEP 69040-000, Brazil; ^3^Laboratório de AIDS e Imunologia Molecular, Instituto Oswaldo Cruz, FIOCRUZ, Rio de Janeiro, RJ CEP 21040-900, Brazil

## Abstract

Virologic failure may occur because of poor treatment adherence and/or viral drug resistance mutations (DRM). In Brazil, the northern region exhibits the worst epidemiological scenarios for the human immunodeficiency virus (HIV). Thus, this study is aimed at investigating the genetic diversity of HIV-1 and DRM in Manaus. The cross-sectional study included people living with HIV on combined antiretroviral therapy and who had experienced virological failure during 2018-2019. Sequencing of the protease/reverse transcriptase (PR/RT) and C2V3 of the viral envelope gp120 (*Env*) regions was analyzed to determine subtypes/variants of HIV-1, DRMs, and tropism. Ninety-two individuals were analyzed in the study. Approximately 72% of them were male and 74% self-declared as heterosexual. Phylogenetic inference (PR/RT-*Env*) showed that most sequences were *B* subtype, followed by BF1 or *BC* mosaic genomes and few F1 and *C* sequences. Among the variants of subtype *B* at PR/RT, 84.3% were pandemic (*B*_PAN_), and 15.7% were Caribbean (*B*_CAR_). The DRMs most frequent were M184I/V (82.9%) for nucleoside reverse transcriptase inhibitors (NRTI), K103N/S (63.4%) for nonnucleoside reverse transcriptase inhibitor (NNRTI), and V82A/L/M (7.3%) for protease inhibitors (PI). DRM analysis depicted high levels of resistance for lamivudine and efavirenz in over 82.9% of individuals; although, low (7.7%) cross-resistance to etravirine was observed. A low level of resistance to protease inhibitors was found and included patients that take atazanavir/ritonavir (16.6%) and lopinavir (11.1%), which confirms that these antiretrovirals can be used—for most individuals. The thymidine analog mutations-2 (TAM-2) resistance pathway was higher in *B*_CAR_ than in *B*_PAN_. Similar results from other Brazilian studies regarding HIV drug resistance were observed; however, we underscore a need for additional studies regarding subtype *B*_CAR_ variants. Molecular epidemiology studies are an important tool for monitoring the prevalence of HIV drug resistance and can influence the public health policies.

The article "High Detection Rate of HIV Drug Resistance Mutations among Patients Who Fail Combined Antiretroviral Therapy in Manaus, Brazil" was published in 2021. Journal: Biomed Res Int.

## 1. Introduction

Since 1996, Brazil has offered free combined antiretroviral therapy(cART) to all people living with HIV/AIDS (PLWHA) regardless of the TCD4+ cell count—and has adopted innovative actions over the years, mainly in primary care [1, 2]. In cART, the drugs used act on different viral targets, and this therapy has brought significant advances in the treatment of PLWHA, such as a fast reduction of the viral load and their more extended maintenance, followed by a significant increase in the TCD4 lymphocyte counts [3, 4]. This has led to better quality of life, with individuals achieving immunological stability and a consequent reduction in the incidence of opportunistic infections and HIV/AIDS-related deaths. Another benefit that stems from the suppression of HIV replication is the reduced possibility of HIV transmission [5, 6].

Treatment failure in HIV therapy can be related to the presence of drug resistance mutations, drug intolerance, and low adherence to therapeutic regimens causing suboptimal ARV dosage, as well as anthropogenic aspects [7, 8] such as physical, psychological, social, or cultural aspects [9]. In addition, the use of ARVs with a low genetic barrier for resistance in the first therapeutic regimen may favor the rapid selection of DRMs [10]. Virological failure is actually defined by the presence of detectable viral load (VL) ≥ 500 copies/ml after at least six months of cART; hence, HIV-1 genotyping is recommended in order to verify the presence of acquired DRMs [11–13]. Depending on the type of DRM, crossresistance to another ARV of the same class could be verified, as reported for thymidine analog mutations (TAMs). TAMs confers crossresistance to nucleoside analogues, potentially affecting first cART regimens, as may prevent the use of another NRTI in subsequent regimens, and could result in the replacement of the ARV class. [14–17].

Despite advances in HIV treatment in Brazil, the North and northeastern regions registered an increase in the AIDS detection rate between 2009 and 2019. In the Amazonas state, detection arose from 31.7 to 34.8 per 100,000 habitants in this period, despite of a 4.5% decrease in the AIDS mortality rate (6.7 to 6.4 per 100,000 habitants). In 2019, Manaus occupied third place in the mortality coefficient rankings (10.5 per 100,000 habitants) and fifth place in AIDS detection rate rankings (54.7 per 100,000 habitants) [18].

The article "High Detection Rate of HIV Drug Resistance Mutations among Patients Who Fail Combined Antiretroviral Therapy in Manaus, Brazil" was published in 2021. Journal: Biomed Res Int.

The genetic diversity of HIV-1 found in the northern region is little distinct from other regions in Brazil [19], characterized mainly by the prevalence of subtype *B* (63-92%), subtype F1 (0-14%), subtype *C* (0-6%), BF1 (4-18%), and *BC* (0-8%) [20–24]. Contrasting to other Brazilian regions, high prevalence of *B*_CAR_ variant (14.4%) was verified in this region [25]. The studies about subtype *B* variants have been focusing in epidemiological aspects; however, the possible impact in the pathogenesis or acquisition of DRM was not investigated.

This problematic epidemiological scenario, along with little data concerning HIV-1 diversity and DRMs in Manaus, led us to investigate these topics in individuals with virological failure ongoing cART schemes.

## 2. Material and Methods

### 2.1. Study Subject Characteristics and Ethical Aspects

This cross-sectional study included 100 individuals with positive HIV-1 serology, who were older than 18 years of age, undergoing antiretroviral therapy for at least six months and presenting virologic failure (viral load ≥ 1000 copies/ml of plasma), receiving a medical request for HIV-1 genotyping following the guidelines of the Brazilian Ministry of Health at the time of the study. All individuals were included in the study and had their samples collected between 2018 and 2019.. All subjects were treated at the Tropical Medicine Foundation-Heitor Vieira Dourado (FMT-HVD), Manaus, Amazonas state, Brazil. Demographic and clinical data were collected using a structured questionnaire. A sample of 4 ml of whole blood was collected by venous pulse, and the samples were processed for plasma separation and stored at -80°C until RNA extraction. The study was approved by the Ethical Review Board, IOC/FIOCRUZ under CAAE 87171018.4.0000.5248 protocol, the FMT-HVD under approval CAAE 87171018.4.3001.0005, and all subjects gave written informed consent in accordance with the Declaration of Helsinki.

### 2.2. RNA and RT-PCR Extraction

Extraction of genetic materials was performed using the QIAamp RNA mini kit (Qiagen, Germany) following the manufacturer's instructions. This was followed by reverse transcription of RNA to obtain cDNA using MMLV enzyme (Invitrogen, Carlsbad, CA) protocol with specific external reverse PCR primers for each gene target.

### 2.3. Amplification, Purification, and Sequencing of PR/RT and C2-V3

The *pol* region was amplified by nested PCR with initial primer G17S (AAAAAGGGCTGTTGTTGGTGGAATGTGGA)/MMRTR6 (TTTTACATTAGTGTGGG) and MMRTR5 (TAAATTTGATATGTCCATTG)/MMRT10 (CAGGCTAATTTTTTAGGGAA) generating a final fragment of 1478 bp (positions 2077-3574 relative to HXB2). For the *env* region, we used the external primers ED5 (ATGGGATCAAAGCCTAAAAGCCATGTG)/ED12 (AGTGCTTCCTGCTGCTCCCAAGAACCCAAG) and ED31(CCTCAGCCATTACACAGGCCTGTCCAAAG)/ED33 (TTACAGTAGAAAAATTCCCCTC) generating a final fragment of 563 bp (positions 6816-7380 relative to HXB2), as described by Delwart et al. and Delatorre et al. [26, 27]. The cycling protocol for both study regions was 94°C for 2 minutes for initial denaturation, followed by 35 cycles of 94°C for 30 seconds, 55°C for 30 seconds, and 72°C for 2 minutes, with a final extension of 10 minutes at 72°C.

The article "High Detection Rate of HIV Drug Resistance Mutations among Patients Who Fail Combined Antiretroviral Therapy in Manaus, Brazil" was published in 2021. Journal: Biomed Res Int.

The amplified PCR products were purified using the Illustra GFX PCR DNA and Gel Band Purification Kit (GE Healthcare, United Kingdom) following the manufacturer's instructions. The products were subsequently subjected to sequencing using ABI BigDye Terminator v.3.1 Cycle Sequencing Ready (Applied Biosystems, United States). The samples were sequenced in the ABI Prism 3130 automatic sequencer (Applied Biosystems).

### 2.4. Sequence Analysis

The sequences were edited using SeqMan software of the DNASTAR 4.0 program and aligned by Clustal W in the MEGA 6.0 program together with corresponding reference sequences of the different HIV-1 subtypes obtained from the Los Alamos database (http://hiv.lanl.gov). The final *pol* (partial PR/RT) and *env* (partial gp120) alignments contained a 1260 nucleotide (nt) (positions 2254-3514 relative to the HXB2) and a 397 nt fragment (positions 6858-7225 relative to the HXB2), respectively.

The phylogenetic analysis was performed based on the neighbor-joining method and the Tamura-Nei substitution model. The bootstrap test with 1,000 replicates was used to estimate the confidence level of the branching on the phylogenetic tree. Possible recombinant sequences were detected via bootscan analysis, which was performed using the Simplot 3.5.1 program. These analyses were performed on a sliding window of 200 nt moving in 10 nt steps. For the characterization of the B_BR_ variant in the C2V3 region, an amino acid sequence was obtained by the translation of the *env* alignment using MEGA, and all sequences showing the GWG motif at the top of loop V3 were considered. The Brazilian HIV-1 B *pol* sequences were aligned using the Clustal W in the MEGA program, with reference B (Pandemic or Caribbean) sequences, and the positions associated with DRMs were removed. The analysis was performed using the maximum likelihood (ML) method in the PhyML program, and the FigTree v1.4.0 program was used for confection and visualization of the phylogenetic trees.

Analysis of PR/RT resistance mutations was performed for each sequence on the Stanford HIV Drug Resistance Database website (http://hivdb.stanford.edu/). All major resistance mutations from the updated list on this site were considered (https://hivdb.stanford.edu/pages/download/resistanceMutations_handout.pdf and https://www.iasusa.org/resources/hiv-drug-resistance-mutations/). The susceptibility of each sequence to the ARV was also determined using the HIVdb Program from the Stanford HIV Drug Resistance Database. However, concerning the resistance level to the ARV only the high-level resistance was applied.

The article "High Detection Rate of HIV Drug Resistance Mutations among Patients Who Fail Combined Antiretroviral Therapy in Manaus, Brazil" was published in 2021. Journal: Biomed Res Int.

The genotypic prediction was used to infer the use of CCR5 and/or CXCR4 coreceptors. The prediction was performed based on the amino acid sequence of the V3 region of the gp120 of the envelope of each sequence using the program Geno2pheno (available at https://coreceptor.geno2pheno.org/), with a false positive cut-off rate of 10% according to the European Tropism Test guidelines.

### 2.5. Statistical Analyses

The data were analyzed using the GraphPad Prism software version 5 and the *R* software, with a significance level set at *P* < 0.05. Statistical comparisons between and within groups were made using Fisher's exact test, the Mann–Whitney test, and the Kruskal-Wallis test when appropriate.

## 3. Results

### 3.1. Epidemiological and Clinical Data

Of the 100 individuals enrolled in the study, we were able to amplifiy 95% at the PR/RT region and to sequence 92% of them. From those 92 individuals, approximately, 72% were male, with an average age of 40 (31-46) years, and approximately, 95% were residents of Manaus, the capital of the Amazonas state. Regarding sexual orientation, 74% declared themselves heterosexual, 19% as homosexual, and 6% as bisexual. The median viral load (log) was 4.4 (IQR 4-5), and the median CD4+ count was 168 cell/mm^3^ (IQR 50.5-342.5) at the time of sample collection. The patients from this cohort presented a mean of six years (IQR 4-7) receiving cATR, 57.6% of them were receiving their first treatment, and 42.4% had already undergone treatment changes (TARV). From the 92 (PR/RT) analyzed individuals, only 78 (84.8%) sequences were determined in the envelope region. Thus, according to the phylogenetic inference of the combined *pol* (RT/PR) and *env* regions together, it was possible to classify these 78 HIV-1 (*pol/env*) sequences as 68.5% subtype *B*/*B*, F1/F1 (1.1%), and *C*/*C* (1.1%), and 14.1%were mosaic genomes, for which 13% BF1 and 1.1% *BC*. However, for the remaining 14 sequences (15.2%) obtained only in the *pol* region, 14.2% were subtype *B*, and 1% was subtype *C*. Regarding the HIV-1 subtype *B* variants, 84.3% were classified as pandemic and 15.7% as Caribbean in the *pol* region, and 5.1% were Brazilian variants (*B*_BR_) in *env*. The bioinformatic analyses were able to predict that the viral tropism found in the sequences of the env region demonstrated that about the majority (66.7%) of the 78 studied individuals sequenced at *env* region had the R5 virus at the time of the sample collection.

The article "High Detection Rate of HIV Drug Resistance Mutations among Patients Who Fail Combined Antiretroviral Therapy in Manaus, Brazil" was published in 2021. Journal: Biomed Res Int.

Among the 92 studied individuals, DRMs were observed in 82 sequences (89%), from those 91.5% presented DRMs associated with NRTI (*n* = 75) and 84.1% with NNRTI (*n* = 69) (Figure 1). All patients were taking NRTIs at the time the genotyping test was done, with 3TC being used by 92.6% of the individuals (*n* = 76/82) and TDF by 84.1% (*n* = 69/82). Concerning NNRTIs, all individuals had already used EFV; however, only 63.4% (n =52/82) were currently using this ARV at the collection time (Table 1). The most frequently detected DRMs were M184I/V (68/82; 82.9%), K70E/R (16/82; 19.5%), and T215F/Y (17/82; 20.7%) to NRTI and K103N/S (51/82; 62.1%), P225H (15/82; 18.2%), and V106A/I/M (11/82; 13.4%) to NNRTI (Figure 1). Thymidine analog mutations (TAM) were detected in 35.4% of the individuals [17.1% (14/82) TAM-1 (including M41L, L210W, and T215Y) and 20.7% (17/82) TAM-2 (including D67N, K70R, T215F, and K219Q/E)].

Only half of the individuals had used PI (*n* = 46/82), only 17% of individuals presented DRMs associated with protease inhibitors (*n* = 14), and the most frequent mutations were V82A/L/M (6/82; 7.3%) and I54L/M/V (5/82; 6%), L90M (4/82; 4.8%), and M46L/I (4/82; 4.8%) (Figure 1). ATZ/r was the most ARV used at the time of the genotyping test (23.1%, *n* = 19/82) (Table 1). Concerning the resistance mutations, the most prevalent inter-ARV class combinations were M184/K103 and M184/K103/P225 (12.1% each) and M184/K70/K103 (8.5%). Multidrug resistance mutations were verified in 72% to NNRTI/NRTI, 5% NRTI/PI, and 3% NNRTI/NRTI/PI.

High resistance level to NRTI class was verified in 85.3% (*n* = 70/82), being most of them 82.9% (*n* = 68/82) among those under 3TC use, and the M184I/V mutation was presented in all of them. However, only 6 from those 70 individuals that were taking TDF (8.5%) had high resistance level against TDF, despite its high use (Table 1), in the same way as high resistance level was detected just in 6 from those 46 individuals that were taking PI (13.0%). TDF remained acceptable as for being used for most of the individuals studied (91.5%), as well as the DRV to all individuals (Table 1). In regard to NNRTI, high ARV resistance level was detected in approximately 90.0% of them, representing 64 of those 71 individuals who were taking EFV, and mutations K103N/S (71.8) and P225H (21.1%) were the most prevalent among them. Among those individuals under use of NRTIs, crossover DRM confers high resistance level to abacavir in 47.5% of them, as well as for the 71 individuals under use of NNRTIs, and high resistance of 66.4% was verified to nevirapine, followed to 39.4% to rilpavirine, 19.7% to doravirine, and only 7.7% to etravirine (data not shown).

The article "High Detection Rate of HIV Drug Resistance Mutations among Patients Who Fail Combined Antiretroviral Therapy in Manaus, Brazil" was published in 2021. Journal: Biomed Res Int.

While analyzing the resistance profile of individuals with B_CAR_ and B_PAN_ variants, the heat map showed that the most frequent mutations in subtype *B* variants were M184I/V (NRTI) and K103N/S (NNRTI), and these also presented similar prevalence in both groups (Figure 2(a)). Despite the low frequencies of TAMs in the general group below 20% (Figure 1), when we compared them among *B*_CAR_ and *B*_PAM_, it was possible to observe that the TAM-2 mutational pattern was more present (*P* = 0.0294) in the *B*_CAR_ variants (Figure 2(b)) and TAM-1 in the *B*_PAM_ variants (*P* = 0.1000).

## 4. Discussion

Even though the northern region has presented one of the worst HIV epidemiological scenarios in Brazil in the last few years, there has been scarce surveillance of epidemiological and molecular resistance. In the present study regarding HIV-1 individuals failing cART individuals, the epidemiological data, genetic HIV-1 diversity,, and frequency of DRMs and their ARV used were analyzed. We observed both high prevalence of individuals with virologic failure without DRMs and also elevated frequency of DRMs, which can lead to an increase of TDRM (transmitted DRMs) and in HIV transmission in the region, as has been recently observed [28].

The general male-to-female ratio (M/F) detected was 2.5, in agreement with a 2.3 rate observed in 2018 in Brazil on a national level [18], and in 2011 in the state of Amazonas during the 2001-2012 HIV/AIDS epidemic [29]. Our results show a higher prevalence of heterosexual individuals. This category represents 71% of the study males, in contrast with the 31.4% observed nationally from 2007 to June 2019 in males over 13 years [18] .

Our results show a high prevalence of HIV-1 subtype *B* and a very low presence of subtypes F1 and *C*, as previously reported in other studies in the state of Amazonas [21, 22, 30, 31]. An increased number of HIV BF1 recombinant forms (13%) were verified when compared to other studies based on the *pol* region (4.3%-10%), mainly because of the inclusion of the *env* region in the analysis. Caribbean variants of subtype *Bpol* viruses were detected in the high rate of 15.7% when compared to other Brazilian regions, which goes in agreement with the 22% previously report at the same Amazon region [32]. A low prevalence (5.1%) of the *B*_BR_ variant of HIV-1 subtype *B* (*env*) was observed [33], in contrast with 20-60% found in studies from other regions in the country [34–37].

The article "High Detection Rate of HIV Drug Resistance Mutations among Patients Who Fail Combined Antiretroviral Therapy in Manaus, Brazil" was published in 2021. Journal: Biomed Res Int.

The majority of the patients in our study had T CD4 counts below 200 cells/mm^3^ even when under a longer period of cART. This could be the result of a long virologic failure period until HIV genotyping and ARV replacement and also due to a late arrival of the individuals to care and consequently late HIV diagnosis. This may be demonstrated by the low CD4 count when analyzing the immune status of patients presenting for the first time, where half of patients showed CD4+ T cell counts below 350/mm^3^ and one-third below 200/mm^3^ at the initial HIV diagnosis [38]. These results also indicate a significant advance in the progression of the infection to AIDS in these individuals.

Concerning the viral tropism based in the sequences of the *env* region, we found that about 33% of the viruses presented X4 tropism; when considering only HIV-1 subtype *Benv* (*n* = 66), the X4 virus was verified in 38% of the individuals, which is very similar to previous reports of 40% of subtype *B* virus switching during disease progression [39, 40]. On the other hand, 66.7% of the analyzed samples in our study still had R5 viral tropism and could be eligible for rescue therapies involving the use of maraviroc, as described by Bon et al. [41].

The studied individuals show high prevalence of DRMs associated with to NRTI (91%) and to NNRTI (84%). Other Brazilian studies have documented an increase in NNRTI DRMs over time, as well as the decrease in the rate of DRMs for NRTI [38, 42]. The increase of NNRTI resistance is mainly correlated to the presence of the K103N mutation, which was detected in 71.8% of individuals that use NNRTI, as also previously described [24]. The prevalence of K103N/S in our study (63.4%) was higher than the mean of 40% detected for the five largest Brazilian cities (São Paulo, Rio de Janeiro, Espirito Santo-Southeast region and Bahia and Ceará-Northeast region) and also in Belém, another city in the northern region [24, 38]. An elevated frequency of M184V (75%) was also detected herein, as well as in the study conducted in Belém [24]; this has ranged from 54.4% in São Paulo to 81.2% in Bahia [38]. Despite the low impact of the M184V alone to NRTI resistance, when taken together to other NRTI DRM, an increased level of resistance could be verified as shown in this study and in others [43–45].

A higher prevalence of TAM 1 was verified herein, as well as a lower prevalence of TAM-2, similar to those reported by Lopes et al. in the northern region [24]. It is important to point out that some resistance mutations observed in our and in other cross-sectional studies conducted with individuals failing cART could result from the transmitted virus since, up until now, genotyping prior to the HIV treatment is required only in a few cases, such as for pregnant women in Brazil, for example.

The article "High Detection Rate of HIV Drug Resistance Mutations among Patients Who Fail Combined Antiretroviral Therapy in Manaus, Brazil" was published in 2021. Journal: Biomed Res Int.

We observed high resistance to 3TC and EFV, and we have also demonstrated that the NRTIs (TDF and AZT) still presented high viability of use for most individuals. Due to the presence of mutations, such as L100I, K101P, Y181C, M230L, observed in of individuals failing in the use of EFV, the viability of using ETR in a rescue scheme is reduced for few individuals (data not shown) [46].

The high resistance levels found for these ARVs (3TC > EFV > TDF) reflect their high use and the genetic barrier to resistance of these ARVs [47]. Although some studies suggest that the viability of using first-line ARV drugs may be related to the combination of drugs with a low and/or high genetic barrier, consequently, the choice of drugs with a low barrier may favor the rapid selection of DRMs causing therapeutic failure [10]. The studied group has little experience with PIs, taken together to the fact that boosted PIs have a high genetic barrier, which could explain the low prevalence of major PI mutations observed. Our results demonstrated a high prevalence of NRTI/NNRTI dual class ARV NNRTI over the years in several studies, and resistance to NNRTI and NRTI is the most common forms of TDR [48–50] Due to the increased prevalence of resistance to NRTI and NNRTI-based regimens, ARVs focusing new targets on the HIV replication cycle were developed and implemented at the therapy. On a clinical trial comparing once-daily dolutegravir versus twice-daily raltegravir in antiretroviral-experienced individuals, the superior virological effect was verified in the dolutegravir group [51]. Dolutegravir has a high genetic barrier to resistance, which can be effective for HIV, both for first-line and rescue schemes. The study by Cahn et al. subsidized the World Health Organization to recommend the use of dolutegravir in the first therapeutic regimen since 2016, and it was implemented in Brazil in 2017. After the genotyping performed at the present study, various of the individuals started to use this ARV.

These factors can contribute to the DRM potentiating therapeutic failure and increase HIV transmission and TDRM prevalence in the region. Thus, the clinical and constant viral load monitoring of PLWHA is essential in order to reduce the risk of DRM accumulation and thus rapidly detect therapeutic failure, in order to preserve susceptibility to subsequent therapeutic schemes [15, 52]. However, protease inhibitors remain a good rescue therapy with less than 13% of the associated resistance verified, despite their use in 50% of individuals.

The article "High Detection Rate of HIV Drug Resistance Mutations among Patients Who Fail Combined Antiretroviral Therapy in Manaus, Brazil" was published in 2021. Journal: Biomed Res Int.

No significant epidemiological differences were seen among individuals infected by subtype *B* variants, as previously verified among specific viral subtypes [53, 54]. Our results showed that the TAM-2 pathway was more prevalent in the *B*_CAR_ variants, while TAM-1 was greater in *B*_PAN_, as shown previously in the northern region in blood donors [28]. It is important to point out that the TAM pathway verified could result from the specific use of thymidine analogs used during the treatment of these individuals. However, specific TAMs pathways were verified in some viral subtypes [55, 56], and these pathways are potentially related to the difficulty in achieving viral suppression [57]. However, further studies are needed to corroborate the specific characteristics concerning HIV-1 subtype *B* variants (*B*_CAR_ and *B*_PAN_) detected herein.

## 5. Conclusion

This is the most comprehensive analysis of the molecular epidemiology of HIV-1 and acquired DRMs in Manaus. Herein, we verified a high prevalence of the HIV-1 subtype *B*, a significant difference in the TAM pathway in relation to *B* variants (*B*_CAR_ and *B*_PAN_), as well as an increase in recombinant BF1. We also verified that, despite the high resistance to 3TC and EFV, the low crossresistance of ARV of the same classes may favor rapid replication control after the change of viable ARV. Therefore, HIV-1 surveillance at local sites is essential for understanding the different obstacles for treatment adherence and rapid detection of therapeutic failure. This information will help the National Health Service redirect its strategies to achieve greater HIV/AIDS control.

## Figures and Tables

**Figure 1:** Frequency of HIV-1 drug resistance mutations according to inhibitor class and TAMs detected in 82 individuals. (a) DRM to NRTI: nucleoside reverse transcriptase inhibitors (91.5%, *n* = 75/82). (b) DRM to NNRTI: nonnucleoside reverse transcriptase inhibitor (84.1%, *n* = 69/82). (c) DRM to PI: protease inhibitors (17%, n =14/82). (d) Thymidine analog mutations TAM [TAM-1 (*n* = 14), TAM-2 (*n* = 17)].

**Figure 2:** Comparison of DRMs among subtype *B* variants: *B*_CAR_ (*n* = 13) and *B*_PAN_ (*n* = 61). (a) Heat map of the different classes of antiretroviral drugs: protease inhibitors (PI), nucleoside reverse transcriptase inhibitors (NRTI) and nonnucleoside reverse transcriptase inhibitors (NNRTI), and the frequency of drug-resistant mutations. (b) Profile of mutation pathways associated with thymidine—TAMs (TAM-1 *B*_CAR_ (*n* = 1) and *B*_PAN_ (*n* = 10) and TAM-2 *B*_CAR_ (*n* = 5) and *B*_PAN_ (*n* = 9) between subtype *B* variants). Statistical analysis using the Mann–Whitney test: TAM-1 (*P* = 0.1000) TAM-2 (*P* = 0.0294).

The article "High Detection Rate of HIV Drug Resistance Mutations among Patients Who Fail Combined Antiretroviral Therapy in Manaus, Brazil" was published in 2021. Journal: Biomed Res Int.

**Table 1:** Prevalence of ARV used at any time during treatment and current in use, prevalence of the most prevalent DRMs to each ARV class in relation to the ARV current in use, and percentage of individuals with high ARV resistance related to the ARV used.

ARV	ARV used, *n* (%)	ARV current in use, *n* (%)	Drug resistance mutation, *n* (%)			ARV high resistance level, *n* (%)
			M184I/V	K70E/R	T215F/Y	
Total NRTI	82/82 (100)	82/82 (100)	68/82 (82.9)	16/82 (19.5)	17/82 (20.7)	70/82 (85.3)
3TC	82/82 (100)	76/82 (92.6)				68/82 (82.9)
TDF	70/82 (85.3)	69/82 (84.1)				6/70 (8.5)
AZT	41/82 (50.0)	5/82 (6.0)				9/41 (21.9)
			K103N/S	V106A/I/M	P225H	
Total NNRTI	71/82 (86.5)	48/82 (58.5)	51/71 (71.8)	11/71 (15.4)	15/71 (21.1)	64/71 (90.1)
EFV	71/82 (86.5)	52/82 (63.4)				64/71 (90.1)
			V82A/L/M	I54L/M/V	M46L/I	
Total PI	46/82 (50.0)	26/82 (31.7)	5/46 (10.8)	5/46 (10.8)	4/46 (8.6)	6/46(13.0)
LPV	18/82 (21.9)	1/82 (1.2)				2/18 (11.1)
ATZ/r	24/82 (29.2)	19/82 (23.1)				4/24 (16.6)
DRV	6/82 (7.3)	4/82 (4.8)				0 (0)

ARVs: 3TC: lamivudine; EFV: efavirenz; TDF: tenofovir; AZT: zidovudine; AZT/r: atazanavir/ritonavir; DRV: darunavir; LPV: lopinavir; PI: protease inhibitors. ARV resistance inputted according to high resistance level in the Stanford HIV Drug Resistance database (https://hivdb.stanford.edu/).

## Data Availability

All nucleotide sequences are available from the GenBank database (https://www.ncbi.nlm.nih.gov/genbank/) under accession numbers POL (MW545333-MW545424) and ENV (MW582429-MW582506).

## References

[1] Brasil A. E. H. V., Ministério da Saúde, Secretaria de Vigilância em Saúde, Departamento de DST (2015). *Cuidado integral às pessoas que vivem com HIV pela Atenção Básica Manual para a equipe multiprofissional*.

[2] Brasil A. E. H. V., Ministério da Saúde, Secretaria de Vigilância em Saúde, Departamento de DST (2018). *Agenda Estratégica para ampliação do acesso e cuidado integral das populações-chave em HIV, hepatites virais e outras infecções sexualmente transmissíveis*.

[3] Hoffmann C. J., Schomaker M., Fox M. P. (2013). CD4 count slope and mortality in HIV-infected patients on antiretroviral therapy. *JAIDS Journal of Acquired Immune Deficiency Syndromes*.

[4] Saag M. S., Benson C. A., Gandhi R. T. (2018). Antiretroviral drugs for treatment and prevention of HIV infection in adults. *JAMA*.

[5] Fokam J., Sosso S. M., Yagai B. (2019). Viral suppression in adults, adolescents and children receiving antiretroviral therapy in Cameroon: adolescents at high risk of virological failure in the era of ‘test and treat. *AIDS Research and Therapy*.

The article "High Detection Rate of HIV Drug Resistance Mutations among Patients Who Fail Combined Antiretroviral Therapy in Manaus, Brazil" was published in 2021. Journal: Biomed Res Int.

[6] Cohen M. S., Chen Y. Q., McCauley M. (2016). Antiretroviral therapy for the prevention of HIV-1 transmission. *New England Journal of Medicine*.

[7] Nachega J. B., Marconi V. C., van Zyl G. U. (2011). HIV treatment adherence, drug resistance, virologic failure: evolving concepts. *Infectious Disorders-Drug Targets*.

[8] Yu Y., Luo D., Chen X., Huang Z., Wang M., Xiao S. (2018). Medication adherence to antiretroviral therapy among newly treated people living with HIV. *BMC Public Health*.

[9] Calvetti P. Ü., Giovelli G. R. M., Gauer G. J. C., de Moraes J. F. D. (2014). Psychosocial factors associated with adherence to treatment and quality of life in people living with HIV/AIDS in Brazil. *Jornal Brasileiro de Psiquiatria*.

[10] Katusiime C., Ocama P., Kambugu A. (2014). Basis of selection of first and second line highly active antiretroviral therapy for hiv/aids on genetic barrier to resistance: a literature review. *African Health Sciences*.

[11] Corado A. D. L. G., Bello G., Leão R. A. C., Granja F., Naveca F. G. (2017). HIV-1 genetic diversity and antiretroviral drug resistance among individuals from Roraima state, northern Brazil. *PLoS One*.

[12] Sanguansittianant S., Nooroon N., Phaengchomduan P., Ammaranond P. (2013). Trends in prevalence of HIV-1 drug resistance in Thailand 2009-2010. *Journal of Clinical Laboratory Analysis.*.

[13] Gupta R. K., Hill A., Sawyer A. W. (2009). Virological monitoring and resistance to first-line highly active antiretroviral therapy in adults infected with HIV-1 treated under WHO guidelines: a systematic review and meta-analysis. *The Lancet Infectious Diseases.*.

[14] Brasil A. E. H. V., Ministério da Saúde, Secretaria de Vigilância em Saúde, Departamento de DST (2008). *Recomendações para terapia anti-retroviral em adultos infectados pelo HIV*.

[15] Sigaloff K. C. E., Ramatsebe T., Viana R., de Wit T. F. R., Wallis C. L., Stevens W. S. (2012). Accumulation of HIV drug resistance mutations in patients failing first-line antiretroviral treatment in South Africa. *AIDS Research and Human Retroviruses.*.

[16] Thirunavukarasu D., Udhaya V., Iqbal H. S., Umaarasu T. (2013). Patterns of HIV-1 drug-resistance mutations among patients failing first-line antiretroviral treatment in South India. *Journal of the International Association of Providers of AIDS Care*.

[17] B.M da S.S de em S.D. de D de C.C e I S T (DCCI) (2019). *Brasil, Ministério da Saúde, Secretaria de Vigilância em Saúde, and Departamento de DST, Manual Técnico para Avaliação de Exames de Genotipagem do HIV*.

[18] Brasil A. E. H. V., Ministério da Saúde, Secretaria de Vigilância em Saúde, Departamento de DST (2019). *Boletim Epidemiológico HIV/Aids |2019*.

The article "High Detection Rate of HIV Drug Resistance Mutations among Patients Who Fail Combined Antiretroviral Therapy in Manaus, Brazil" was published in 2021. Journal: Biomed Res Int.

[19] Gräf T., Pinto A. R. (2013). The increasing prevalence of HIV-1 subtype C in southern Brazil and its dispersion through the continent. *Virology*.

[20] Carvalho B. C., Cardoso L. P. V., Damasceno S., Stefani M. M. D. A. (2011). Moderate prevalence of transmitted drug resistance and interiorization of HIV type 1 subtype C in the inland north state of Tocantins, Brazil. *AIDS Research and Human Retroviruses.*.

[21] Cunha L. K. H., Kashima S., Amarante M. F. C. (2012). Distribution of human immunodeficiency virus type 1 subtypes in the state of Amazonas, Brazil, and subtype C identification. *Brazilian Journal of Medical and Biological Research.*.

[22] Da Costa C. M., Costa De Oliveira C. M., Chehuan De Melo Y. F., Delatorre E., Bello G., Couto-Fernandez J. C. (2016). High HIV-1 genetic diversity in patients from northern Brazil. *AIDS Research and Human Retroviruses.*.

[23] Dos Anjos Silva L., Divino F., Da Silva Rêgo M. O. (2016). HIV-1 genetic diversity and transmitted drug resistance in antiretroviral treatment-naive individuals from Amapá state, northern Brazil. *AIDS Research and Human Retroviruses.*.

[24] Lopes C. A. F., Soares M. A., Falci D. R., Sprinz E. (2015). The evolving genotypic profile of HIV-1 mutations related to antiretroviral treatment in the north region of Brazil. *BioMed Research International*.

[25] Divino F., De Corado A. L. G., Naveca F. G., Stefani M. M. A., Bello G. (2016). High prevalence and onward transmission of non-pandemic HIV-1 subtype B clades in northern and northeastern brazilian regions. *PLoS One*.

[26] Delwart E., Shpaer E., Louwagie J. (1993). Genetic relationships determined by a DNA heteroduplex mobility assay: analysis of HIV-1 env genes. *Science*.

[27] Delatorre E., Silva-De-Jesus C., Couto-Fernandez J. C., Pilotto J. H., Morgado M. G. (2017). High HIV-1 diversity and prevalence of transmitted drug resistance among antiretroviral-naive HIV-infected pregnant women from Rio de Janeiro, Brazil. *AIDS Research and Human Retroviruses.*.

[28] Esashika Crispim M. A., da Guarda Reis M. N., Fraiji N., Bello G., Stefani M. M. A. (2019). Detection of human immunodeficiency virus type 1 phylogenetic clusters with multidrug resistance mutations among 2011 to 2017 blood donors from the highly endemic northern Brazilian Amazon. *Transfusion*.

[29] De Oliveira R. D. S. M., Benzaken A. S., Saraceni V., Sabidó M. (2015). Hiv/aids epidemic in the state of amazonas: Characteristics and trends from 2001 to 2012. *Revista da Sociedade Brasileira de Medicina Tropical*.

[30] Crispim M. A. E., Reis M. N. D. G., Abrahim C. (2019). Homogenous HIV-1 subtype B from the Brazilian Amazon with infrequent diverse BF1 recombinants, subtypes F1 and C among blood donors. *PLOS ONE*.

The article "High Detection Rate of HIV Drug Resistance Mutations among Patients Who Fail Combined Antiretroviral Therapy in Manaus, Brazil" was published in 2021. Journal: Biomed Res Int.

[31] De Andrade S. D., Sabidó M., Monteiro W. M., Benzaken A. S., Tanuri A. (2017). Drug resistance in antiretroviral-naive children newly diagnosed with HIV-1 in Manaus, Amazonas. *Journal of Antimicrobial Chemotherapy*.

[32] Vicente A. C. P., Otsuki K., Silva N. B. (2000). The HIV epidemic in the Amazon Basin is driven by prototypic and recombinant HIV-1 subtypes B and F. *Journal of Acquired Immune Deficiency Syndromes*.

[33] Morgado M. G., Guimarães M. L., Gripp C. B. G. (1998). Molecular epidemiology of HIV-1 in Brazil: high prevalence of HIV-1 subtype B and identification of an HIV-1 subtype D infection in the city of Rio de Janeiro, Brazil. *Journal of Acquired Immune Deficiency Syndromes and Human Retrovirology*.

[34] Pimentel V. F., Morgado M. G., Bello G. (2013). Temporal trends and molecular epidemiology of HIV type 1 infection in Rio de Janeiro, Brazil. *AIDS Research and Human Retroviruses.*.

[35] Potts K. E., Kalish M. L., Lott T. (1993). Genetic heterogeneity of the V3 region of the HIV-1 envelope glycoprotein in Brazil. *AIDS*.

[36] MORGADO M. G., SABINO E. C., SHPAER E. G. (1994). V3 region polymorphisms in HIV-1 from Brazil: prevalence of subtype B strains divergent from North American/European prototype and detection of subtype F. *AIDS Research and Human Retroviruses*.

[37] Junqueira D. M., de Medeiros R. M., Ferreira Leite T. C. N. (2013). Detection of the B″-GWGR variant in the southernmost region of Brazil: unveiling the complexity of the human immunodeficiency virus-1 subtype B epidemic. *Memorias do Instituto Oswaldo Cruz*.

[38] Diaz R. S., Inocêncio L. A., Sucupira M. C. A. (2015). The virological and immunological characteristics of the HIV-1-infected population in Brazil: from initial diagnosis to impact of antiretroviral use. *PLoS One*.

[39] Mild M., Kvist A., Esbjörnsson J., Karlsson I., Fenyö E. M., Medstrand Patrik P. (2010). Differences in molecular evolution between switch (R5 to R5X4/X4-tropic) and non-switch (R5-tropic only) HIV-1 populations during infection. *Infection, Genetics and Evolution*.

[40] Tscherning C., Alaeus A., Fredriksson R. (1998). Differences in chemokine coreceptor usage between genetic subtypes of HIV-1. *Virology*.

[41] Bon I., Clò A., Borderi M. (2013). Prevalence of R5 strains in multi-treated HIV subjects and impact of new regimens including maraviroc in a selected group of patients with CCR5-tropic HIV-1 infection. *International Journal of Infectious Diseases*.

[42] Duani H., Aleixo A. W., Tupinambás U. (2017). Trends and predictors of HIV-1 acquired drug resistance in Minas Gerais, Brazil: 2002–2012. *Brazilian Journal of Infectious Diseases*.

The article "High Detection Rate of HIV Drug Resistance Mutations among Patients Who Fail Combined Antiretroviral Therapy in Manaus, Brazil" was published in 2021. Journal: Biomed Res Int.

[43] Harrigan P. R., Stone C., Griffin P. (2000). Resistance profile of the human immunodeficiency virus type 1 reverse transcriptase inhibitor abacavir (1592U89) after monotherapy and combination therapy. *The Journal of Infectious Diseases*.

[44] Bacheler L., Jeffrey S., Hanna G. (2001). Genotypic correlates of phenotypic resistance to efavirenz in virus isolates from patients failing nonnucleoside reverse transcriptase inhibitor therapy. *Journal of Virology*.

[45] Melikian G. L., Rhee S. Y., Varghese V. (2014). Non-nucleoside reverse transcriptase inhibitor (NNRTI) cross-resistance: implications for preclinical evaluation of novel NNRTIs and clinical genotypic resistance testing. *Journal of Antimicrobial Chemotherapy*.

[46] Madruga J. V., Cahn P., Grinsztejn B. (2007). Efficacy and safety of TMC125 (etravirine) in treatment-experienced HIV-1-infected patients in DUET-1: 24-week results from a randomised, double-blind, placebo-controlled trial. *Lancet*.

[47] Tang M. W., Shafer R. W. (2012). HIV-1 Antiretroviral Resistance. *Drugs*.

[48] Rhee S. Y., Blanco J. L., Jordan M. R. (2015). Geographic and temporal trends in the molecular epidemiology and genetic mechanisms of transmitted HIV-1 drug resistance: an individual-patient- and sequence-level meta-analysis. *PLoS Medicine*.

[49] Gupta R. K., Jordan M. R., Sultan B. J. (2012). Global trends in antiretroviral resistance in treatment-naive individuals with HIV after rollout of antiretroviral treatment in resource-limited settings: a global collaborative study and meta-regression analysis. *The Lancet.*.

[50] Wensing A. M., Calvez V., Ceccherini-Silberstein F. (2019). 2019 update of the drug resistance mutations in HIV-1. *Topics in antiviral medicine.*.

[51] Cahn P., Pozniak A. L., Mingrone H. (2013). Dolutegravir versus raltegravir in antiretroviral-experienced, integrase- inhibitor-naive adults with HIV: week 48 results from the randomised, double- blind, non-inferiority SAILING study. *The Lancet*.

[52] De Luca A., Sidumo Z. J., Zanelli G. (2017). Accumulation of HIV-1 drug resistance in patients on a standard thymidine analogue-based first line antiretroviral therapy after virological failure: implications for the activity of next-line regimens from a longitudinal study in Mozambique. *BMC Infectious Diseases*.

[53] Venner C. M., Nankya I., Kyeyune F. (2016). Infecting HIV-1 subtype predicts disease progression in women of sub-Saharan Africa. *eBioMedicine*.

[54] Kiwanuka N., Laeyendecker O., Robb M. (2008). Effect of human immunodeficiency virus type 1 (HIV-1) subtype on disease progression in persons from Rakai, Uganda, with incident HIV-1 infection. *The Journal of Infectious Diseases.*.

The article "High Detection Rate of HIV Drug Resistance Mutations among Patients Who Fail Combined Antiretroviral Therapy in Manaus, Brazil" was published in 2021. Journal: Biomed Res Int.

[55] Novitsky V., Wester C. W., DeGruttola V. (2007). The reverse transcriptase 67N 70R 215Y genotype is the predominant TAM pathway associated with virologic failure among HIV type 1C-infected adults treated with ZDV/ddI-containing HAART in southern Africa. *AIDS Research and Human Retroviruses.*.

[56] Marcelin A. G., Delaugerre C., Wirden M. (2004). Thymidine analogue reverse transcriptase inhibitors resistance mutations profiles and association to other nucleoside reverse transcriptase inhibitors resistance mutations observed in the context of virological failure. *Journal of Medical Virology*.

[57] Hanna G. J., Johnson V. A., Kuritzkes D. R. (2000). Patterns of resistance mutations selected by treatment of human immunodeficiency virus type 1 infection with zidovudine, didanosine, and nevirapine. *The Journal of Infectious Diseases*.

